# The prevalence and clinicopathological features of breast cancer patients with hepatitis B virus infection in China

**DOI:** 10.18632/oncotarget.15305

**Published:** 2017-02-13

**Authors:** He Wu, Chunxia Zhao, Vishnu Prasad Adhikari, Linjie Lu, Jianbo Huang, Yuxian Wei, Qingqing Luo, Wei Dai, Yutuan Wu, Xin Li, Kainan Wu, Ling-Quan Kong

**Affiliations:** ^1^ Department of Endocrine and Breast Surgery, The First Affiliated Hospital of Chongqing Medical University, Chongqing 400016, China; ^2^ Department of Thyroid and Breast Surgery, Liuzhou People's Hospital, Liuzhou 545006, Guangxi, China

**Keywords:** hepatitis B surface antigens, breast neoplasms, pathology, hepatitis B infection, epidemiology

## Abstract

We performed a case-control study to investigate the prevalence and clinicopathological features of breast cancer patients with hepatitis B virus (HBV) infection in China. The clinical data for 2,796 female patients with newly diagnosed, primary breast cancer were evaluated. A total of 234 breast cancer patients with HBV infection (the case group; positive for hepatitis B surface antigen [HBsAg]) and 444 breast cancer patients without HBV infection (the control group; negative for HBsAg, hepatitis B surface antibody, hepatitis B envelope antigen, hepatitis B envelope antibody, and hepatitis B core antibody) were selected for study. Analysis of the clinicopathological features revealed that the metastatic axillary lymph node ratio was lower in the case group than the control group, as was the proportion of patients with pathological T stage ≥T2. No differences in the expression levels of estrogen receptor, progesterone receptor, human epidermal growth factor receptor 2, p53, or Ki67 were observed between the case and control groups. These data indicate that the rate of HBV infection is high among female breast cancer patients in China, and that HBsAg-positive breast cancer patients were generally diagnosed at an earlier stage and had fewer lymph node metastases.

## INTRODUCTION

Breast cancer is the most commonly diagnosed cancer among women in the United States. It accounts for approximately 29% of all new cancer diagnoses in women [1]. Among Chinese women, breast cancer is most frequently diagnosed cancer between the ages of 30 and 59 years, and it is the leading cause of cancer-related death in women less than 45 years of age [2]. An estimated 2 billion individuals worldwide are infected with the hepatitis B virus (HBV). Of these individuals, approximately 350–400 million have chronic HBV infection [3]. In China, every surgical patient undergoes routine testing for HBV serological markers to prevent cross-infection during preoperative preparation. Although the universal HBV immunization program for newborns that was initiated in 1992 has decreased the prevalence of hepatitis B surface antigen (HBsAg) carriers from 9.8% in 1992 to 7.18% in 2006, HBV still has a significant socioeconomic burden in developing countries including China [4].

HBV can damage hepatocytes, which are important for estrogen inactivation in the liver. This can result in an increase in the estrogen concentration in the blood in patients with HBV infection. Abnormally high estrogen levels are associated with an increased incidence of certain types of cancer, particularly those of the breast [5]. Several studies have shown that increased exposure to free estrogen as a consequence of chronic liver dysfunction may promote breast cancer [6, 7]. Breastfeeding has been evaluated as a potential source of mother-to-child transmission of HBV (either through HBsAg in breast milk or through exposure to infected blood via nipple abrasions), suggesting that HBV may persist in the breast ducts or in mammary glandular cells [8]. Estrogen receptor α (ERα) mediates transcriptional downregulation of NTCP, which is a major entry receptor for HBV [9]. Interestingly, estrogen decreases viral load and inhibits the immune system from attacking the virus, suggesting a strong association between HBV infection and breast cancer. Although a direct correlation between breast cancer and HBV infection has not yet been established, the HBV X protein (can immortalize mammary gland epithelial cells and may be a critical factor in carcinogenesis [10]. High levels of HBV X-interacting protein (HBXIP) were associated with breast cancer progression. Therefore, it could be a valuable prognostic marker and/or therapeutic target in breast cancer [11]. HBXIP expression was predominantly observed in breast tumor tissue compared to adjacent normal tissue. Additionally, HBXIP was shown to play a critical oncogenic role in breast cancer cells [11, 12]. In this study, we aimed to perform a case-control study to investigate the prevalence and clinicopathological features of breast cancer patients with HBV infection in China.

## RESULTS

Of 2,796 patients with primary breast cancer, 234 (8.3%) also had HBV. Of these patients, 1,415 (50.6%) were positive for HBsAb and 1,698 (60.7%) were positive for HbcAb. The results of the comparative analysis of the clinicopathological features of breast cancer patients in the case and control groups is shown in Table 1. The metastatic axillary lymph node ratio in breast cancer patients with HBV infection was significantly lower than that of the control group (33.1 vs. 42.8 %, P = 0.04). The proportion of patients with pathological T stage ≥T2, in breast cancer patients with HBV infection was also significantly lower in the case than in the control group (≥ T2: 48% vs. 58.7%, P = 0.01). No statistically significant differences were observed in family history of malignancy, tumor location, pathological T stage, histological type, histological grade, or ER, PR, HER2, p53, and Ki67 expression.

**Table 1:** Comparative analysis of the clinicopathological features of breast cancer patients in the case and control groups

	Case group		Control group		P
	N	%	N	%	
Family history of malignancy					
Yes	20	9.0	34	8.0	
No	202	91.0	390	92.0	0.66
Location					
Left	129	58.1	222	50.5	
Right	93	41.9	218	49.5	0.06
Pathological T stage					
Tis	1	0.5	4	0.9	
T1	104	52.0	173	40.9	
T2	86	43.0	217	51.3	
T3	9	4.5	29	6.9	0.06
T1	104	52.0	173	41.3	
≥ T2	95	48.0	246	58.7	0.01
Histological grade❈					
Grade 1	1	0.9	10	4.4	
Grade 2	95	83.3	186	82.3	
Grade 3	18	15.8	30	13.3	0.19
Histological type❈					
Invasive	140	87.5	272	85.0	
*In situ*	9	5.6	13	4.1	
Other	11	6.9	35	10.9	0.29
Number of lymph node metastases❈					
0	107	66.9	183	57.2	
> 0	53	33.1	137	42.8	0.04
Cancer embolus❈					
Yes	1	0.6	5	1.6	
No	159	99.4	315	98.4	0.35
ER					
Positive	130	66.3	268	70.0	
Negative	66	33.7	115	30.0	0.20
PR					
Positive	115	58.7	232	60.3	
Negative	81	41.3	153	39.7	0.71
Her-2					
Positive	45	29.8	106	70.2	
Negative	88	31.0	196	69.0	0.79
p53					
Positive	137	71.0	274	72.1	
Negative	56	29.0	106	27.9	0.78
Ki67					
< 14 %	66	34.2	126	32.9	
≥ 14 %	127	65.8	257	67.1	0.75

❈Denotes the 160 breast cancer patients with HBV infection who underwent surgery immediately after diagnosis (case group). These data were compared to those of 320 breast cancer patients who were negative for HBV serological markers (HBsAg, HBsAb, HBeAg, HBeAb, and HBcAb) and who underwent surgery immediately after diagnosis).

## DISCUSSION

Several previous studies have demonstrated a link between viral infections and breast cancer. For example, the presence of viral-like sequences (e.g. Epstein-Barr virus, human papillomavirus, and mouse mammary tumor virus) has been demonstrated in human breast cancer tissue as well as in some normal breast tissue and breastmilk epithelial cells [13, 14]. An estimated 2 billion people are thought to have been infected with HBV worldwide, although the prevalence of HBsAg carriers in China had decreased to approximately 7.18% in 2006 [4]. Chinese women generally have a low risk of breast cancer. However, the incidence of breast cancer is increasing in China [2]. Thus, the relationship between HBV infection and breast cancer should be further investigated.

Here, we analyzed 2,796 Chinese women with primary breast cancer. Of these patients, 234 (8.3%) were positive for HBsAg and 507 (18.1%) were negative for HBV serological markers (HBsAg, HBsAb, HBeAg, HBeAb, and HBcAb). The incidence of HBV infection among the breast cancer patients in our study population was 8.3%, which is higher than that the incidence reported for the Chinese population in 2006 (7.18%) [4]. Finally, the prevalence of viral hepatitis in men is higher than in women [15]. This is also true for acute hepatitis [16], which likely has a lower incidence among female HBsAg carriers than was reported previously (7.18% in China approximately 10 years ago).

We performed a comparative assessment of the clinicopathological features of breast cancer patients with HBV infection. The case group consisted of patients who were positive for HBsAg (222 patients, average age of 48.8 years), and the control group consists of patients were negative for HBV serological markers (HBsAg, HBsAb, HBeAg, HBeAb and HBcAb; 444 patients, average age of 48.7 years). There were no significant differences in family history of malignancy, tumor location, histological type, histological grade, or the presence of cancer emboli. We conclude that family history of malignancy did not impact breast cancer incidence in our population, which may explain the higher incidence of breast cancer patients with HBV infection.

Although there were no significant differences in family history of malignancy, tumor location, pathological T stage, histological type, histological grade, or ER, PR, HER2, p5,3 and Ki67 expression between the case and control groups, the metastatic axillary lymph node ratio, and ratio of tumor size ≥ T2 were significantly lower in the case than in the control groups, suggesting that breast cancer patients who are positive for HBsAg at the time of initial diagnosis are less likely to have axillary lymph node metastasis and more likely to have smaller tumors. These findings are not consistent with the results of a study of the relationship between breast cancer and diabetes [17]. Interestingly, breast cancer patients with diabetes were more likely to have axillary lymph node metastasis, and advanced pathological T stage and grade [17]. Our data suggest that HBV infection may protect against tumor development and axillary lymph node metastasis in breast cancer. A recent study indicated one algorithm (IHC4, 4 IHC markers) did not provide statistically significant prognostic information between years 5 and 10, with the exception of nodal status and tumor size [18]. We speculate that breast cancer patients with HBV infection may have a better prognosis than those who do not have HBV.

A meta-analysis demonstrated that type 2 diabetes significantly increases the incidence of breast cancer and may be an independent prognostic factor for the risk of recurrence and metastasis. These results could explain why HBV infection is also an independent prognostic factor for breast cancer [19]. The authors suggest that the high rate of advanced tumor histological grade and lymph node metastasis in diabetic breast cancer patients may be associated with insulin resistance. Hyperinsulinemia could enhance the activity of insulin-like growth factor and promote tumor growth, since tumor cells consume large amounts of glucose, and high glucose levels drive tumor growth [20]. Based on previous studies of the relationship between estrogen/ER and HBV replication [21], and the mechanisms responsible for insulin resistance, we think that HBV may reduce the levels of estrogen and/or the ER thereby suppressing tumor growth in patients with HBV infection.

In summary, we observed a high incidence of HBV infection in breast cancer patients in China. Breast cancer patients who were positive for HBsAg at the time of initial diagnosis were generally diagnosed at an earlier stage and had a reduced incidence of lymph node metastasis. Our results should be validated in future studies with larger sample sizes.

## MATERIALS AND METHODS

### Study population

The study was performed at the Breast Cancer Center of Chongqing at The First Affiliated Hospital of Chongqing Medical University. It was approved by the Ethics Committee of The First Affiliated Hospital of Chongqing Medical University. There were 2,796 female patients with primary breast cancer who received surgical treatment at the Breast Cancer Center of Chongqing between June 2012 and December 2015. This cancer center is one of the largest in southwest China (covering a population of 31.4 million residents who live in an approximately 82,402.95 km^2^ area). In China, every surgical patient must undergo routine examination of HBV serological markers to prevent cross-infection. The clinical data for 2,796 female patients who were newly diagnosed with primary breast cancer and who had consecutive data for HBV serological markers available in electronic medical records were screened based on HBV status. We found that 234 of these breast cancer patients (8.3%) had HBV. HBV was diagnosed based on HBsAg positivity [22].

We performed a case-control study consisting of 222 female breast cancer patients with HBV infection (the case group, positive for HBsAg). This group included 160 patients who underwent surgery immediately after diagnosis and 62 patients who received neoadjuvant chemotherapy prior to surgery. The control group consisted of 444 breast cancer patients who did not have HBV (negative for the following serological markers: hepatitis B surface antigen [HBsAg], hepatitis B surface antibody [HBsAb], hepatitis B envelope antigen [HBeAg], hepatitis B envelop antibody [HBeAb], and hepatitis B core antibody [HBcAb]). This group included 320 breast cancer patients who underwent surgery immediately after diagnosis and 124 patients who received neoadjuvant chemotherapy prior to surgery. We performed a comparative analysis of the clinicopathological features of all patients in the case and control groups.

### Data collection

Data including age, family history of malignancy, tumor location, and treatment with adjuvant therapies were obtained from patient medical records. A total of 222 female breast cancer patients who were HBsAg-positive with an average age of 48.8 years were selected for the case group. Controls were randomly selected and age-matched (within 5 years), with an average age of 48.7. The control group consisted of 444 breast cancer patients with negative HBV markers The age of the patients between the case and control groups shows no significant differences, *p* = 0.824). The pathological T stage, histological grade, and lymph node status were determined using the American Joint Committee on Cancer Staging Manual (6^th^ edition). Histological data regarding estrogen receptor (ER), progesterone receptor (PR), human epidermal growth factor receptor 2 (HER2), p53, and Ki67 expression were obtained from pathology reports generated at the Pathology Center of Chongqing at Chongqing Medical University. Core needle biopsy results were obtained for patients who received neoadjuvant chemotherapy prior to surgery, and post-surgical gross specimen biopsy results were obtained for patients who underwent surgery immediately after diagnosis (preoperative core needle or intraoperative frozen biopsies). HER-2 status was initially assessed using either immunohistochemistry (IHC) or fluorescence *in situ* hybridization (FISH). Both analyses were performed by the Pathology Center of Chongqing, Chongqing Medical University. HER-2 positive patients were FISH positive (HER-2 amplification) or IHC 3+. HER-2 negative patients were FISH negative (no HER-2 amplification) or IHC 0–1+. Patients were classified as borderline if they were IHC 2+ only (no FISH results available).

### Statistical analysis

Clinicopathological features were compared between the case and control groups using chi-squared tests. A P < 0.05 was considered statistically significant. The SPSS software (Version 19.0) was used to analyze differences in ER, PR, HER2, p53, and Ki67 expression between groups.
